The article "Seasonal and Temperature-Associated Increases in Gram-Negative Bacterial Bloodstream Infections among Hospitalized Patients" was published in 2011. Journal: PLoS One.

# Seasonal and Temperature-Associated Increases in Gram-Negative Bacterial Bloodstream Infections among Hospitalized Patients

**DOI:** 10.1371/journal.pone.0025298

**Published:** 2011-09-26

**Authors:** Michael R. Eber, Michelle Shardell, Marin L. Schweizer, Ramanan Laxminarayan, Eli N. Perencevich

**Affiliations:** 1 Center for Disease Dynamics, Economics and Policy, Washington, D.C., United States of America; 2 University of Maryland School of Medicine, Baltimore, Maryland, United States of America; 3 University of Iowa Carver School of Medicine, Iowa City, Iowa, United States of America; 4 Princeton Environmental Institute, Princeton, New Jersey, United States of America; 5 Iowa City VA Medical Center, Iowa City, Iowa, United States of America; Los Angeles Biomedical Research Institute, United States of America

## Abstract

**Background:**

Knowledge of seasonal trends in hospital-associated infection incidence may improve surveillance and help guide the design and evaluation of infection prevention interventions. We estimated seasonal variation in the frequencies of inpatient bloodstream infections (BSIs) caused by common bacterial pathogens and examined associations of monthly BSI frequencies with ambient outdoor temperature, precipitation, and humidity levels.

**Methods:**

A database containing blood cultures from 132 U.S. hospitals collected between January 1999 and September 2006 was assembled. The database included monthly counts of inpatient blood cultures positive for several clinically important Gram-negative bacteria (*Acinetobacter* spp, *Escherichia coli*, *Klebsiella pneumoniae*, and *Pseudomonas aeruginosa*) and Gram-positive bacteria (*Enterococcus* spp and *Staphylococcus aureus*). Monthly mean temperature, total precipitation, and mean relative humidity in the postal ZIP codes of participating hospitals were obtained from national meteorological databases.

**Results:**

A total of 211,697 inpatient BSIs were reported during 9,423 hospital-months. Adjusting for long-term trends, BSIs caused by each Gram-negative organism examined were more frequent in summer months compared with winter months, with increases ranging from 12.2% for *E. coli* (95% CI 9.2–15.4) to 51.8% for *Acinetobacter* (95% CI 41.1–63.2). Summer season was associated with 8.7% fewer *Enterococcus* BSIs (95% CI 11.0–5.8) and no significant change in *S. aureus* BSI frequency relative to winter. Independent of season, monthly humidity, monthly precipitation, and long-term trends, each 5.6°C (10°F) rise in mean monthly temperature corresponded to increases in Gram-negative bacterial BSI frequencies ranging between 3.5% for *E. coli* (95% CI 2.1–4.9) to 10.8% for *Acinetobacter* (95% CI 6.9–14.7). The same rise in mean monthly temperature corresponded to an increase of 2.2% in *S. aureus* BSI frequency (95% CI 1.3–3.2) but no significant change in *Enterococcus* BSI frequency.

The article "Seasonal and Temperature-Associated Increases in Gram-Negative Bacterial Bloodstream Infections among Hospitalized Patients" was published in 2011. Journal: PLoS One.

**Conclusions:**

Summer season and higher mean monthly outdoor temperature are associated with substantially increased frequency of BSIs, particularly among clinically important Gram-negative bacteria.

## Introduction

Seasonal variation in the incidence of human infection can influence diagnosis and empiric treatment and has the potential to guide both the design and the evaluation of infection prevention interventions. The importance of seasonal variation in community-associated infection incidence is well recognized, particularly for influenza [1]. Each year, the emergence of seasonal influenza in cold, winter months drives heightened public health initiatives to prevent and control transmission, including surveillance for infections, vaccination of at-risk populations, and educational outreach to health care workers and the public at large.

Certain hospital-associated pathogens, particularly Gram-negative bacteria, are increasingly recognized as exhibiting seasonal trends in infection incidence [2]–[5]. However, prior studies examining seasonality of hospital-associated infections have been limited by analysis of small numbers of infections [3]–[5]. Existing studies have also been limited by their inability to assess independent associations of infections with meteorological elements that may be driving these seasonal trends [2], [5]. Confirmation of seasonal patterns and the factors behind these trends will facilitate infection prevention and control by focusing public health efforts. Knowledge of seasonal trends will also allow for improved designs of quasi-experimental (before-after) studies, which are frequently used when assessing infection prevention interventions. Without adjusting for seasonal trends, these studies could be biased by seasonal fluctuations in infection incidence unrelated to the policies or interventions under investigation [6].

The objective of this study was to evaluate seasonal changes in the frequencies of bloodstream infections (BSIs) caused by Gram-negative and Gram-positive bacterial pathogens using a large, nationally representative database of clinical cultures collected from inpatients in the United States. This study focused on blood cultures to ensure that positive cultures reflected infections and not merely colonizing organisms [7]. Potential meteorological drivers of seasonal trends [3], [4], [8] were also examined by assessing independent associations between monthly frequencies of infections and local outdoor temperature, precipitation, and humidity levels.

The article "Seasonal and Temperature-Associated Increases in Gram-Negative Bacterial Bloodstream Infections among Hospitalized Patients" was published in 2011. Journal: PLoS One.

## Methods

### Data sources

The microbiology data source for the analysis was The Surveillance Network-USA database (TSN), a nationally representative database of clinical cultures collected from hospital patients [9]. Inpatient blood cultures positive for Gram-positive bacteria (*Enterococcus* spp and *Staphylococcus aureus*) or Gram-negative bacteria (*Acinetobacter* spp, *Escherichia coli*, *Klebsiella pneumoniae*, and *Pseudomonas aeruginosa*) that were reported between January 1999 and September 2006 were included in the analysis. To avoid bias from duplicate clinical cultures taken from the same patient, only one randomly selected culture per patient per pathogen was retained during each clinical episode. For each pathogen, a clinical episode was defined as a period when consecutive cultures from the same patient were taken ≤30 days apart [10].

To assess the relationship between weather variation and infection incidence, monthly climate data corresponding to the ZIP code of each included hospital were collected from the National Climatic Data Center's Climate Data Online system. Daily data on mean temperature, total precipitation, and mean dew point temperature (a marker of humidity) were aggregated to the monthly level. Because dew point temperature was highly correlated with temperature in our data (r = 0.95), we did not include this variable along with temperature in statistical analyses. Instead, the Magnus-Tetens approximation was used to estimate mean monthly relative humidity using temperature and dew point temperature data [11], [12]. Resulting relative humidity estimates were weakly correlated with temperature (r = −0.10) and other explanatory variables and were therefore included in the multivariate analyses.

### Statistical analysis

Overdispersed Poisson mixed-effects regression models of monthly aggregated hospital-level BSI counts were used to perform a time-series analysis to estimate percentage changes in infections in spring (April–June), summer (July–September), and autumn (October–December) compared with winter (January–March). Random intercepts accounted for within-hospital correlation. Natural cubic splines with 7 degrees of freedom were used to adjust for long-term time trends. The models were adjusted for the nine U.S. Census Bureau regional divisions to account for regional variation in BSIs. An additional set of models was constructed similarly, including indicator terms for calendar month instead of indicators for season to examine monthly trends in BSI frequencies.

To examine associations between BSIs and meteorological variables, two additional Poisson mixed-effects time-series regression models were fit for each organism. One model estimated effects of changes in weather variables (temperature, humidity, and precipitation) over all seasons and adjusted for season, census regional division, and long-term time trends using natural cubic splines (with 7 degrees of freedom). Another season-specific model included weather-by-season interaction terms to examine associations of weather variables with BSI within each season (e.g., warmer vs. cooler summers). Temperature, humidity, and precipitation were modeled as continuous variables and were included as linear terms in both models.

The article "Seasonal and Temperature-Associated Increases in Gram-Negative Bacterial Bloodstream Infections among Hospitalized Patients" was published in 2011. Journal: PLoS One.

Data analysis was conducted using Stata version 10.0 and R software version 2.7.1. Statistical significance was set at the 95% level.

### Sensitivity analysis

Estimates of changes in infection frequency in different seasons might not accurately reflect changes in incidence rates of infection if numbers of infections vary with seasonal changes in hospital populations. Information on the patient populations of institutions submitting to the clinical culture database was unavailable. Therefore, we examined the potential bias caused by seasonal variation in the national number of hospital admissions in the United States over the analysis period by calculating national estimates of the mean yearly number of hospital admissions in each season over the analysis period using the Healthcare Cost and Utilization Project Nationwide Inpatient Sample database [13].

### Ethics

Institutional review board approval was not needed because this study did not involve analysis of human subjects as defined in 45 C.F.R. § 46.102(f). An exception from review was obtained from the University of Iowa Institutional Review Board. The study involved analysis of an existing database of specimens in which subjects could not be identified, either directly or through identifiers linked to subjects. For these reasons, written consent by patients for information to be stored in the database was not required.

## Results

A total of 211,697 blood cultures of the selected organisms were reported over 9,423 hospital-months. Hospitals reporting blood cultures represented all nine U.S. census regional divisions (Table 1). The South Atlantic region contributed the greatest number of hospital-months of data (1,928); the New England region contributed the fewest (294).

**Table 1:** Distribution of hospitals, by U.S. region.

Region	Hospitals	Hospital-months
East North Central	17	1,194
East South Central	9	644
Mid-Atlantic	18	1,080
Mountain	8	664
New England	4	294
Pacific	22	1,687
South Atlantic	26	1,928
West North Central	13	779
West South Central	15	1,153
United States	132	9,423

Of the organisms examined, *S. aureus* was cultured most frequently, accounting for a median of 976 BSIs (interquartile range, 828–1,037) per month over all reporting hospitals (Table 2). *Acinetobacter* was cultured the least frequently, accounting for a median of 67 BSIs (interquartile range, 51–81) per month over all reporting hospitals.

The article "Seasonal and Temperature-Associated Increases in Gram-Negative Bacterial Bloodstream Infections among Hospitalized Patients" was published in 2011. Journal: PLoS One.

**Table 2:** Adjusted percentage change in inpatient BSI frequency in spring, summer, and autumn compared with winter.*

Infecting organism	Median total BSIs reported per month (IQR)	Adjusted percentage change in BSI frequency (95% CI) compared with winter		
		Spring	Summer	Autumn
Gram-negative bacteria				
*Acinetobacter* spp	67 (51, 81)	18.1 (9.5 to 27.5)	51.8 (41.1 to 63.2)	32.3 (22.6 to 42.8)
*E. coli*	472 (404, 509)	8.5 (5.6 to 11.5)	12.2 (9.2 to 15.4)	5.2 (2.2 to 8.2)
*K. pneumoniae*	227 (198, 258)	10.4 (6.1 to 15.0)	28.6 (23.7 to 33.7)	12.8 (8.4 to 17.5)
*P. aeruginosa*	159 (138, 183)	6.4 (1.5 to 11.7)	28.1 (22.3 to 34.1)	14.2 (8.8 to 19.9)
Gram-positive bacteria				
*Enterococcus* spp	430 (362, 485)	−5.5 (−8.1 to −2.8)	−8.5 (−11.0 to −5.8)	−6.9 (−9.5 to −4.2)
*S. aureus*	976 (828, 1037)	−3.2 (−5.0 to −1.4)	−1.7 (−3.6 to 0.1)	−1.3 (−3.2 to 0.6)

BSI = bloodstream infection; CI = confidence interval; IQR = interquartile range.

*Percentage change = 100×(relative BSI frequency−1). Estimated using Poisson mixed-effects regression models with random intercepts to account for within-site correlation, natural cubic splines (with 7 degrees of freedom) to adjust for long-term trends, and adjustment for census region.

### Seasonal trends in bacterial bloodstream infections

After adjusting for long-term trends, BSIs caused by each of the Gram-negative organisms examined were most frequent in summer months (Table 2 and Figure 1). *Acinetobacter* exhibited the greatest seasonal variation in infection frequency, displaying a 51.8% (95% CI 41.1–63.2) increase in BSI frequency in summer months compared with winter months. *E. coli* BSIs exhibited the most modest summer peaks among Gram-negative bacterial BSIs; *E. coli* BSIs were 12.2% (95% CI 9.2–15.4) more frequent in summer relative to winter. The Gram-positive organisms examined, by contrast, did not exhibit summer peaks in BSI frequency. *Enterococc*us BSIs were 8.5% (95% CI 5.8–11.0) less frequent during summer compared with winter, and *S. aureus* BSI frequency was not significantly different.

**Figure 1:** Point estimates indicate monthly mean BSI counts based on regression models. Solid trend lines plot adjusted monthly means on natural cubic splines of calendar month (3 degrees of freedom for *P. aeruginosa*, 2 degrees of freedom for other organisms). Dotted lines indicate 95% confidence intervals.

The article "Seasonal and Temperature-Associated Increases in Gram-Negative Bacterial Bloodstream Infections among Hospitalized Patients" was published in 2011. Journal: PLoS One.

### Associations of meteorological elements with bacterial bloodstream infections

Mean monthly outdoor temperature was positively associated with frequencies of BSIs caused by Gram-negative bacteria and *S. aureus* (Table 3). An increase in mean monthly temperature of 5.6°C (10°F) corresponded to independent increases in *Acinetobacter*, *E. coli*, *K. pneumonia*, and *P. aeruginosa* BSI frequencies of 10.8% (95% CI 6.9–14.7), 3.5% (95% CI 2.1–4.9), 8.0% (95% CI 6.0–10.1), and 7.5% (95% CI 5.1–10.0), respectively. For *S. aureus*, an increase in temperature of 5.6°C (10°F) was associated with an adjusted increase of 2.2% (95% CI 1.3–3.2) in frequency of BSIs. A significant association with temperature was not observed for *Enterococcus* BSIs.

**Table 3:** Associations of mean monthly temperature with inpatient BSI frequencies over all seasons and within seasons.*

Infecting organism	Adjusted percentage change in BSI frequency (95% CI) per 5.6°C (10°F) increase in monthly temperature				
	Associations over all seasons†	Associations within seasons‡			
		Winter	Spring	Summer	Fall
Gram-negative bacteria					
*Acinetobacter* spp	10.8 (6.9 to 14.7)	9.5 (4.0 to 15.0)	13.2 (8.2 to 18.3)	8.0 (3.7 to 12.5)	11.1 (6.3 to 16.1)
*E. coli*	3.5 (2.1 to 4.9)	4.5 (2.7 to 6.3)	4.6 (3.0 to 6.3)	1.5 (−0.1 to 3.0)	3.1 (1.4 to 4.8)
*K. pneumoniae*	8.0 (6.0 to 10.1)	9.2 (6.5 to 12.0)	6.4 (3.9 to 8.9)	5.4 (3.2 to 7.7)	8.5 (6.0 to 11.1)
*P. aeruginosa*	7.5 (5.1 to 10.0)	6.4 (3.3 to 9.6)	6.5 (3.4 to 9.6)	5.0 (2.2 to 7.8)	9.6 (6.6 to 12.7)
Gram-positive bacteria					
*Enterococcus* spp	0.3 (−1.1 to 1.7)	1.2 (−0.7 to 3.0)	0.5 (−1.3 to 2.4)	−1.5 (−3.2 to 0.1)	−0.7 (−2.5 to 1.1)
*S. aureus*	2.2 (1.3 to 3.2)	3.4 (2.1 to 4.6)	2.2 (1.1 to 3.4)	−0.3 (−1.4 to 0.7)	2.0 (0.8 to 3.2)

BSI = bloodstream infection; CI = confidence interval.

*Estimated using Poisson mixed-effects regression models with random intercepts to account for within-site correlation, natural cubic splines (7 degrees of freedom) to control for long-term trends, and adjustments for census region. Linear terms for both total monthly precipitation and mean relative humidity were included.

† Model included controls for season.

‡ Models included season and weather-by-season interaction term.

Table 3 also shows adjusted associations of temperature and bacterial BSI frequencies separately within each season. In winter, spring, and fall, higher temperature was positively and significantly associated with infections caused by each Gram-negative organism examined and by *S. aureus*. In summer, higher temperature was positively and significantly associated with infections caused by each Gram-negative pathogen except *E. coli*.

The article "Seasonal and Temperature-Associated Increases in Gram-Negative Bacterial Bloodstream Infections among Hospitalized Patients" was published in 2011. Journal: PLoS One.

For most organisms analyzed, neither monthly precipitation levels nor humidity levels were significantly associated with increased frequency of BSIs in multivariate analyses. For *S. aureus* and *E. coli*, a one-inch increase in monthly precipitation was associated with a 0.3% lower (95% CI 0.1–0.6) frequency of BSIs and a 0.5% lower (95% CI 0.1–1.0) frequency of BSIs, respectively. Increased relative humidity was associated with increased frequency of *P. aeruginosa* BSI (5.8% per 10% relative humidity increase; 95% CI 3.1–8.6).

### National estimates of seasonal trends in hospital admissions

Estimates from the Nationwide Inpatient Sample database of the national average inpatient census over the analysis period showed that winter was the season with the greatest mean number of admissions per year. Compared with winter, there were 2.5%, 1.8%, and 2.5% fewer admissions in spring, summer, and fall, respectively. If hospital admissions in the study sample followed national trends in seasonal variation, estimates of the percentage changes in infections in spring, summer, and fall months compared with winter months presented in Table 2 would slightly underestimate changes in incidence rates of infection.

## Discussion

This eight-year study of 132 hospitals in the United States showed substantial summer increases in the frequencies of inpatient bloodstream infections caused by clinically important Gram-negative bacteria, particularly *Acinetobacter* spp. Summer peaks in BSI frequencies were not observed among Gram-positive bacteria. Within seasons, higher outdoor temperature was consistently associated with increased frequency of BSIs caused by Gram-negative bacteria, with the associations of greatest magnitude observed for organisms that exhibited the greatest relative summer increases in BSI frequency. Increased temperature was associated with a relatively modest but statistically significant increase in *S. aureus* BSI frequency but no significant change in *Enterococcus* BSI frequency. These results suggest that variation in temperature, both within and between seasons, may drive changes in the incidence of bacterial BSIs.

Several previous studies have reported peaks in infections caused by Gram-negative bacteria in warmer months. A multicenter study of *Acinetobacter* infections in United States ICU patients between 1987 and 1996 found that infection rates were more than 50% higher in warmer months compared with colder months [2]. Unlike the present study, this previous study was limited to one organism and did not assess associations between infections and potential meteorological drivers of seasonal changes. Smaller studies have also reported seasonal variation in Gram-negative bacterial infections. A recent study of inpatients at one tertiary-care hospital observed higher incidences of several Gram-negative bacterial infections, but not Gram-positive bacterial infections, in summer months [4]. Another recent study examined *Klebsiella* spp bloodstream infections at four hospitals on different continents and observed higher infection rates in warmer months irrespective of calendar season [3]. The results of the present, large study confirm and expand the results of previous analyses.

The article "Seasonal and Temperature-Associated Increases in Gram-Negative Bacterial Bloodstream Infections among Hospitalized Patients" was published in 2011. Journal: PLoS One.

There are several potential explanations for the observed association of Gram-negative BSI frequency with outdoor temperature levels. First, higher temperatures may facilitate increased growth of bacteria in the environment, which may, in turn, increase colonization of humans [3], [14]. Previous reports have indicated that many organisms in the hospital environment contributing to nosocomial infections originate from the inflow of organisms carried by patients and health care workers [15]. Mechanisms of bacterial growth and optimal growth temperatures vary by organism [16], which may explain the observed differences in associations between organisms. Second, evidence suggests that elevated temperatures may be associated with increased virulence of Gram-negative bacteria [17], [18]. The lipid A moiety of lipopolysaccharide, which forms the outer monolayer of the outermost membrane of most Gram-negative bacteria, is regulated by environmental conditions and is known to modulate virulence in Gram-negative organisms [17], [18]. Thus, it is possible that temperature may modulate the virulence of Gram-negative bacteria, contributing to increases in infection incidence in warmer periods.

Knowledge that certain clinically important infections are substantially more frequent in summer months may facilitate improved surveillance for and empiric treatment of infections. For example, the value of undertaking additional warm-season surveillance of patients or environmental sources, such as municipal drinking water, to prevent infections caused by Gram-negative bacteria might be investigated further. Of note, such interventions might have limited value if important antibiotic-resistant phenotypes of Gram-negative organisms exhibited different seasonal trends. However, in our data, the subset of *Acinetobacter* blood cultures reported to be resistant to imipenem, an indicator of multidrug resistance [19], exhibited a 72.3% (95% CI 32.3–124.6) increase in infection frequency in summer relative to winter based on regression analysis adjusting for long-term trends (data not shown). Imipenem-resistant *P. aeruginosa* blood cultures exhibited a 33.4% (95% CI 17.0–52.1) increase in frequency in summer compared with winter (data not shown).

The article "Seasonal and Temperature-Associated Increases in Gram-Negative Bacterial Bloodstream Infections among Hospitalized Patients" was published in 2011. Journal: PLoS One.

Knowledge of seasonal trends in infections should also improve the design and evaluation of longitudinal, quasi-experimental (before-after) studies. Epidemiologic investigations that seek to determine independent risk factors for certain infections and/or seek to evaluate the potential effects of infection prevention interventions using quasi-experimental study designs should control for seasonal variation in infection incidences [6]. For example, if a quasi-experimental infection control study sought to determine the effect of an active-surveillance program on the incidence of Gram-negative bacterial infections, ignoring the effect of seasonal variation on infection incidences could bias the findings.

Although the most consistent and largest associations with season and temperature were observed for the Gram-negative organisms, a significant association was observed between mean monthly temperature and *S. aureus* BSI frequency. Additional research is warranted to examine whether this relationship could contribute to differences in *S. aureus* infection rates observed across locations, such as differences between Southern and Northern Europe. Although a seasonal association was not demonstrated in our results, previous reports have suggested that certain *S. aureus* infections, including methicillin-resistant *S. aureus* (MRSA) infections, may fluctuate with season. For example, using data from a large Rhode Island hospital, Mermel and colleagues noted seasonality among community-associated MRSA infections in summer and autumn, and seasonality in pediatric hospital-associated MRSA infections [20].

This study has several limitations. First, the analysis is limited in its ability to measure infection incidence because we were unable to measure the populations over time of each institution submitting culture data. It is possible that because of seasonal differences in hospital populations, seasonal differences in infection frequencies might not reflect differences of similar magnitude in incidence rates of infection. However, we explored seasonal trends in the number of hospital admissions nationally, which suggested that our results should slightly underestimate increases in incidence rates of infection in summer compared with winter. Thus, our estimates are likely conservative. Second, although the database captured cultures from all regions of the United States, it is not completely representative of the United States, and certain regions, such as New England, are underrepresented. The specific hospital sample selection may influence the seasonal and temperature results reported. Third, potential non-weather-related seasonal factors, such as intern inexperience with infection control methods and obtaining clinical cultures at different frequencies in summer, could affect the reported results [4]. However, the different seasonal trends observed for Gram-positive organisms and Gram-negative organisms provide *prima facie* evidence that the observed seasonality of Gram-negative infections is related to the organisms and not to potentially confounding factors that would be expected to affect the observed frequencies of infections uniformly across organisms. Fourth, the present analysis was not able to identify nosocomial infections explicitly. Previous single-center studies have not found significant differences in seasonality of nosocomial infections compared with community-associated infections [4]. Fifth, we were not able to examine the relative contributions of environmental conditions within hospitals [21], [22], compared with environmental conditions external to hospitals, in predicting infection incidences. Future studies should examine the modifiable contribution of indoor environmental conditions in predicting changes in infection frequency, which has particularly important implications for hospital decision makers. Finally, a broader set of inpatient infections caused by Gram-negative organisms may exhibit summer peaks in infection incidence [2], [4]. This study did not directly examine seasonality of non-bloodstream infections; however, the mechanisms by which environmental factors drive changes in infection frequency may be similar for other types of hospital-associated infections caused by the same pathogens.

The article "Seasonal and Temperature-Associated Increases in Gram-Negative Bacterial Bloodstream Infections among Hospitalized Patients" was published in 2011. Journal: PLoS One.

In conclusion, we reported substantial increases in the frequencies of bloodstream infections due to clinically important Gram-negative organisms in summer months. These increases, as well as variations in infection frequencies within seasons, appear to be associated with elevated monthly outdoor temperatures. The seasonal trends reported may be used to inform infection prevention and should be considered in the design and evaluation of longitudinal quasi-experimental studies of infection prevention interventions. Furthermore, if the underlying mechanisms of the temperature associations are identified, these findings could inform the global climate change debate.
